The article "Snapback-Free Reverse-Conducting SOI LIGBT with an Integrated Self-Biased MOSFET" was published in 2022. Journal: Nanoscale Res Lett.

# Snapback-Free Reverse-Conducting SOI LIGBT with an Integrated Self-Biased MOSFET

**DOI:** 10.1186/s11671-022-03685-5

**Published:** 2022-04-18

**Authors:** Kemeng Yang, Jie Wei, Kaiwei Dai, Zhen Ma, Congcong Li, Xiaorong Luo

**Affiliations:** The State Key Laboratory of Electronic Thin Films and Integrated Devices, University of Electronic Science and Technology of China, Chengdu, 610054 China

**Keywords:** Lateral insulated gate bipolar transistor (LIGBT), Snapback effect, Reverse conducting, Area-efficient

## Abstract

A novel snapback-free RC-LIGBT with integrated self-biased N-MOSFET is proposed and investigated by simulation. The device features an integrated self-biased N-MOSFET(ISM) on the anode active region. One side of the ISM is shorted to the P + anode electrode of RC-LIGBT and the other side is connected to the N + anode via a floating ohmic contact. The adaptively turn-on/off of the ISM contributes to improve the static and dynamic performance of the ISM RC-LIGBT. In the forward-state, due to the off-state of the ISM, the snapback could be effectively suppressed without requiring extra device area compared to the SSA (separated shorted anode) and STA (segmented trenches in the anode) LIGBTs. In the reverse conduction, the ISM is turned on and the parasitic NPN in the ISM is punched through, which provides a current path for the reverse current. Meanwhile, during the turn-off and reverse recovery states, the ISM turns on, providing a rapid electron extraction path. Thus, a superior tradeoff between the on-state voltage drop (*V*_on_) and turnoff loss (*E*_off_) as well as an improved reverse recovery characteristic can be obtained. Compared to the STA device, the proposed ISM RC-LIGBT reduces *E*_off_ by 21.5% without snapback. Its reverse recovery charge is reduced by 53.7%/58.6% compared to that of the SSA LIGBT with *L*_b_ = 40/60 μm at the same *V*_on_. Due to the prominent static and dynamic characteristic, the power loss of ISM RC-LIGBT in a completed switching cycle is reduced.

## Introduction

The lateral insulated gate bipolar transistor (LIGBT) on silicon-on-insulator (SOI) technology is an attractive device to be used in three-phase single chip inverter ICs due to its low on-state voltage (*V*_on_) under high current density and easy integration [1–3]. However, the unidirectional switch characteristic requires the conventional LIGBT connecting in anti-parallel with a diode to conduct the reverse current, which introduces stray inductance and the extra chip area [4, 5]. The usage of the shorted anode (SA) LIGBT, instead of the conventional LIGBT with an antiparallel diode in the switching modules, proves to be an effective method to address drawbacks as motioned above [6–8]. Meanwhile, the introduced N + anode in the SA LIGBT also provides an electron extraction path and avoids the long current tail during turn-off, resulting in a small turn-off loss. However, the introduced N + anode also makes the SA LIGBT suffers from the undesirable snapback effect, which may lead to the device reliability problems.

The article "Snapback-Free Reverse-Conducting SOI LIGBT with an Integrated Self-Biased MOSFET" was published in 2022. Journal: Nanoscale Res Lett.

To suppress the snapback effect, many structures are proposed. The separated SA LIGBT (SSA LIGBT) alleviates the snapback by increasing the space and the distributed resistance between the P + anode and N + anode [9], while it needs a large device area to effectively eliminate the snapback effect. The segmented trenches in the anode (STA) LIGBT [10] and trench barrier shorted anode (TBSA) LIGBT [11] decrease the distance between N + and P + anode by implementing deep oxide trenches at anode side, while the process is difficult and also increases the cost. Multi-gates devices show better performance by controlling the anode gate, but it needs complex controlling circuits [12–15]. Integrating a diode in the LIGBT to realize reverse conduction and suppress snapback is a smart method, yet the schottky barrier diode makes the performance of the device to be influenced by the temperature [16].

In this paper, a novel area-efficient and snapback-free RC-LIGBT with Integrated Self-biased MOSFET (ISM) is proposed and its mechanism is investigated by Sentaurus TCAD tools. The implemented models include HighFieldSaturation mobility, Philips unified mobility, Auger recombination, Enormal mobility, Shockley–Read–Hall recombination, and Lackner avalanche generation. The adaptively turned-on/off ISM leads to the snapback-free forward conduction characteristic, a decreased turn-off loss and a superior reverse recovery characteristic. As a result, the proposed device performs a reduced power loss in a completed switching cycle.

## Device Structure and Mechanism

Figure 1a shows the schematic of the proposed RC LIGBT featured an Integrated Self-biased MOSFET. The integrated MOSFET on the top of the anode active region does not need extra device area. One side of the ISM is shorted to the P + anode and the other side is connected to the N + anode via a floating ohmic contact (FOC), as illustrated in Fig. 1b. It is worth noting that the ISM is self-adaptively turned on/off according to the operation status of the RC-LIGBT. As Fig. 1b denoted, *N*_P_ and *L*_P_ are the doping concentration and length of the P region in ISM, respectively. *t*_OX_ is the thickness of the oxide of ISM. *N*_A_ and *N*_N_ are the doping concentration of P + anode and N-buffer, respectively.

**Fig. 1:** **a** Schematic cross section of the ISM RC-LIGBT; **b** zoomed-in schematic cross section of the anode side; schematic cross section of **c** SSA LIGBT and **d** STA LIGBT

Figure 2 gives the operation mechanism of the ISM RC-LIGBT. There is a parasitic open base NPN in the ISM. Both the ISM and NPN will be discussed. Figure 2a, b show the equivalent circuits of ISM RC-LIGBT at Forward/ Reverse Conducting (FC/RC) states, respectively. It reveals that the operation state of the ISM influences the current path. Figure 2c summarizes the states of the ISM and the open base NPN under following four operation states of the ISM RC-LIGBT: forward conduction, reverse conduction, turn-off and reverse recovery. Figure 2 reveals that the states of the ISM and NPN influence the current path. The parasitic NPN turns on by depleting the base region.

The article "Snapback-Free Reverse-Conducting SOI LIGBT with an Integrated Self-Biased MOSFET" was published in 2022. Journal: Nanoscale Res Lett.

**Fig. 2:** Equivalent circuit of the ISM RC-IGBT for **a** FC state and **b** RC state. **c** States of the ISM under different operation states of LIGBT. Here, *V*_PN_ is the built-in potential of P+/N-buffer junction, *V*_T_ is the threshold voltage of the self-biased MOS

In the forward conduction, the ISM and the parasitic NPN are in off-state when the P + / N-buffer junction turns on. In this case, the current flowlines only derive from the P + anode and the device operates in the bipolar mode, as shown in the Fig. 3a. When the *N*_P_ vale is too small, the P region in the ISM is fully depleted and then electrons are swept through the NPN, as shown in Fig. 3b. The current flowlines go through the NPN region, while the P + /N-buffer junction is still in off-state. In this case, the device is in unipolar mode at the initial forward-conducting state, resulting in snapback, which should be avoided. Thus, a high *N*_P_ is profited to suppress snapback effect. However, a high *N*_P_ makes the ISM hard to turn on and weakens the effect of reducing the turn-off loss and reverse recovery charges, which will be discussed in detail later.

**Fig. 3:** Current flowlines in the forward-conducting state for the ISM RC-LIGBT (*L*_P_ = 0.8 μm, *t*_OX_ = 50 nm, @*V*_AK_ = 1 V): **a** *N*_P_ = 5 × 10^15^ cm^−3^; **b** *N*_P_ = 1 × 10^14^ cm^−3^

In the reverse conduction, the ISM and parasitic NPN are adaptively turned on, providing a reverse conducting path and realize RC. Figure 4 shows the reverse-conducting current flowlines. With the increasing |*V*_AK_|, the ISM undergoes three cases as follows: the expansion of depleted region near the channel and the ISM is in off-state, as shown in Fig. 4a; inversion layer in the ISM is formed and the ISM turns on, as shown in Fig. 4b; and both the ISM and the parasitic NPN are in on-state, as shown in Fig. 4c. The turned-on ISM is vital to realize the reverse-conducting for the RC-LIGBT.

The article "Snapback-Free Reverse-Conducting SOI LIGBT with an Integrated Self-Biased MOSFET" was published in 2022. Journal: Nanoscale Res Lett.

**Fig. 4:** Current flowlines in the reverse-conducting state for the ISM RC-LIGBT (*N*_P_ = 1 × 10^16^ cm^−3^, *L*_P_ = 0.8 μm, *t*_OX_ = 50 nm): **a** *V*_AK_ =  − 0.5 V; **b** *V*_AK_ =  − 1.5 V; **c** *V*_AK_ =  − 4 V

During turn-off and reverse recovery period, excess electrons in the neutral region drift to the P + anode which is a barrier for electrons (holes can be rapidly swept to the cathode by the high electric field of the depletion region), and thus its extraction mainly determines the speed of turn-off and reverse recovery. For the proposed device, the large voltage between anode and cathode triggers the parasitic NPN in the ISM and then electrons are swept through the NPN, providing an additional electron extracting path. As a result, the extra electrons stored in the drift region could be rapidly removed and the ISM LIGBT achieves a low turn-off loss and reverse recovery charges.

## Results and Discussion

In order to verify the operation mechanisms and advantages of the proposed ISM RC LIGBT, SSA/STA LIGBTs and the conventional LIGBTs with an anti-parallel diode are also simulated and compared. The optimized parameters for each device in simulation are listed in Table 1. All devices are designed with a forward blocking capability of 300 V.

**Table 1:** Key Parameters for LIGBTs

Parameters	ISM	CON	SSA	STA
SOI layer thickness, *t*_s_ (μm)	6	6	6	6
Buried oxide thickness, *t*_BOX_ (μm)	3	3	3	3
N-drift doping, *N*_d_ (× 10^15^ cm^−3^)	3.6	3.6	3.6	3.6
N-drift length, *L*_d_ (μm)	30	30	30	30
N-buffer doping, *N*_buffer_ (× 10^17^ cm^−3^)	2	2	2	2
Doping of the N + region in the ISM (× 10^18^ cm^−3^)	1	–	–	–
Length of the N + region in the ISM (μm)	0.6	–	–	–
Spacing between trenches, *S*_T_ (μm)	–	–	–	0.5
Distance between P + and N + anode, *L*_b_ (μm)	1	–	40/60	5

Figure 5 shows the conduction characteristics of different type LIGBTs. In the forward conduction, the ISM RC-LIGBT with optimal *N*_P_ and *L*_P_ can eliminate snapback without increasing the *V*_on_. For the SSA LIGBT, even though the *L*_b_ achieves 40 μm, the snapback effect still exists and its *V*_on_ is much larger than that of the ISM RC-LIGBT. The STA LIGBT could suppress the snapback, but it still degenerates the *J*_A_ and the *V*_on_ is larger than ISM RC-LIGBT. The proposed structure features a better forward conduction characteristic than the other LIGBTs with a shorted anode. At the reverse-conducting state, the *V*_F_ = 1.8 V for the ISM LIGBT at *J*_A_ = 100 A/cm^2^ is higher than 1.62 V of SSA LIGBT with *L*_b_ = 60 μm, because the RC current path from the cathode to anode in the ISM RC-LIGBT flows through a diode and an NMOS in series.

The article "Snapback-Free Reverse-Conducting SOI LIGBT with an Integrated Self-Biased MOSFET" was published in 2022. Journal: Nanoscale Res Lett.

**Fig. 5:** Comparison of conduction characteristics for ISM, STA, SSA LIGBTs and Con. LIGBT& diode. *S*_T_ is the spacing between the segmented trenches for the STA LIGBT. *L*_b_ is the distance between N-buffer and separated N + anode for the SSA LIGBT. For ISM device, *N*_P_ = 1.5 × 10^15^ cm^−3^, *L*_P_ = 0.8 μm

Figure 6a depicts the influence of key parameters of *N*_P_, *L*_P_ and *t*_OX_ on conduction characteristics for ISM RC-IGBT. With the increasing *N*_P_ or *L*_P_, the snapback effect is weakened and even eliminated as shown by the red and blue lines. Whereas, the devices with *t*_OX_ = 50 and 100 nm exhibit the same forward conduction characteristics owing to the hardly turned-on ISM at FC state. Thus, the forward-conducting characteristic of ISM RC-LIGBT mainly depends on the state of the parasitic NPN. To suppress the snapback, the P + /N-buffer junction should be turned on earlier than the parasitic NPN, namely

1 $$V_{{{\text{PN}}}} \le V_{{{\text{PT}}}}$$

where *V*_PT_ is the punch-through voltage of parasitic NPN in the ISM. Taking formulas of *V*_PN_ and *V*_PT_ [17] into Eq. (1), the parameters of the ISM should satisfy

2 $$N_{{\text{P}}} L_{{\text{P}}}^{2} \ge \frac{{2\varepsilon_{{\text{S}}} kT}}{{q^{{2}} }}\ln \left( {\frac{{N_{{\text{A}}} N_{{\text{N}}} }}{{n_{i}^{2} }}} \right)$$

where *n*_i_ is the intrinsic carrier concentration, *q* is the electronic charge, *ε*_S_ is dielectric constant of Si, *k* is the Boltzmann constant, and* T* is the absolute temperature. In the RC state, with the decreasing *N*_P_, *L*_P_ or *t*_OX_, the diode-mode forward voltage (*V*_F_) of ISM RC-LIGBT is reduced. Both the punched-through NPN and the turned-on ISM contribute to the increase in the reverse current.

**Fig. 6:** **a** Influence of the *N*_P_, *L*_P_ and *t*_OX_ on conduction characteristics. **b** 3-D graph of influence of the *N*_P_ and *L*_P_ on the ∆*V*_SB_

Figure 6b illustrates the influence of the *N*_P_ and *L*_P_ on the ∆*V*_SB_ and denotes the snapback-free region. It is worth noting that the optimal value of *N*_P_ for FC and RC state is the opposite trend. Thus, the optimized relationship of *N*_P_ and *L*_P_ is obtained when the equal sign is taken in Eq. (2), namely the boundary of snapback-free region in Fig. 6b. Figure 6b also reveals that the optimal relation of *N*_P_ and *L*_P_ obtained by simulation is consistent with the calculated results of the model. Therefore, the model could provide a guidance to select the appropriate values of the *N*_P_, *L*_P_, *N*_A_ and *N*_N_ so as to achieve a snapback-free device.

Figure 7a gives the turn-off waveforms of different LIGBTs. The ISM RC-LIGBT turns off the fastest and SSA LIGBT has the longest turn-off time due to the extra *L*_S_ region. To investigate the turn-off mechanism of ISM RC-LIGBT, Fig. 7b gives the electron current flowlines at point A in Fig. 7a. It reveals that the parasitic NPN in the ISM is adaptively turned on. It provides an additional path to rapidly remove the electrons from the drift region. This is constructive to reduce the *E*_off_. In terms of the SSA and STA LIGBT, the long or narrow electron extraction path weakens the effect of reducing *E*_off_. Thus, the ISM RC-IGBT features a better *E*_off_–*V*_on_ tradeoff performance than SSA and STA LIGBTs, as shown in Fig. 8. The *E*_off_ of ISM RC-LIGBT is reduced by 21.5% compared to that of the STA LIGBT with the same *V*_on_ at *J*_A_ = 100 A/cm^2^. Compared with the SSA LIGBT with *L*_b_ = 40/60 μm, ISM LIGBT reduces *V*_on_ by 13.3%/20.8% at the same *E*_off_, because ISM RC-LIGBT does not occupy additional area to eliminate the snapback. Even at higher turn-off current density of 200 A/cm^2^, the ISM LIGBT still exhibits better tradeoff performance than SSA and STA LIGBTs, as illustrated in Fig. 8b. Figure 9 gives the impact of *N*_P_ and *L*_P_ on the tradeoff between *V*_on_ and *E*_off_. The ISM RC-LIGBT with small *N*_P_ and *L*_P_ performs the smallest *E*_off_ due to the easy turn-on ISM and parasitic NPN. However, the small *N*_P_ and *L*_P_ leads to the snapback effect as denoted in Fig. 6. In order to make a balance between the above-mentioned characteristics, *N*_P_ and *L*_P_ are chosen to be 1 × 10^15^ cm^−3^ and 0.8 μm, respectively.

The article "Snapback-Free Reverse-Conducting SOI LIGBT with an Integrated Self-Biased MOSFET" was published in 2022. Journal: Nanoscale Res Lett.

**Fig. 7:** **a** Turn-off waveforms under clamped inductive load with *L*_C_ = 4µH, *L*_S_ = 1nH, *R*_G_ = 10 Ω, *V*_bus_ = 150 V, *V*_on_ = 1.5 V. **b** Electron current flowlines for the ISM RC-LIGBT at anode side [at point A in (**a**)]

**Fig. 8:** *E*_off_ versus *V*_on_ for different LIGBTs: **a** *J*_A_ = 100A/cm^2^ and **b** *J*_A_ = 200A/cm^2^

**Fig. 9:** *E*_off_ versus *V*_on_ for the ISM RC-LIGBT with different *N*_P_ and *L*_P_ at *J*_A_ = 100A/cm^2^

Figure 10 compares the reverse recovery characteristics of the ISM RC-LIGBT, SSA LIGBT and the conventional LIGBT with an anti-parallel diode. The test circuit is shown in Fig. 10a. In Fig. 10b, the reverse recovery charge *Q*_rr_ of the ISM RC-LIGBT is 13.3% lower than that of the conventional LIGBT with an antiparallel diode, due to its 30% reduced reverse recovery peak current. Compared to the SSA LIGBT (*L*_b_ = 40/60 μm) device, *Q*_rr_ of ISM RC-LIGBT is reduced by 53.7%/58.6%. Figure 10c gives the electron distribution in the *x*-dimension from *t*_1_ to *t*_4_ period (denoted in Fig. 10b). Compared to the SSA LIGBT, the ISM RC-LIGBT extracts the electrons more quickly, since the punched-through parasitic NPN in the ISM contributes to a fast electron extraction from drift region. In addition, the ISM RC-LIGBT does not introduce extra electron storage region *L*_b_ as the SSA LIGBT does. Therefore, ISM RC-LIGBT exhibits a better reverse recovery performance than the SSA LIGBT.

The article "Snapback-Free Reverse-Conducting SOI LIGBT with an Integrated Self-Biased MOSFET" was published in 2022. Journal: Nanoscale Res Lett.

**Fig. 10:** Reverse recovery characteristics of the ISM RC-LIGBT, SSA LIGBT and the conventional LIGBT with an anti-parallel diode: **a** circuit diagram for reverse recovery (*L*_C_ = 1mH, *L*_S_ = 1nH, *R*_G_ = 25Ω, *V*_bus_ = 200 V, *V*_on_ = 2 V); **b** reverse recovery waveforms; **c** electron concentration distribution along *y* = 4 μm

In order to investigate the characteristic of ISM RC-LIGBT, the waveforms in a complete on/off switching cycle are compared for the ISM RC-LIGBT, STA and SSA LIGBT (*L*_b_ = 60 μm) in Fig. 11. The circuit diagram is shown in Fig. 10a and the device under test is RC-IGBT2. During the turn-on period, the current overshoot is caused by the reverse recovery of RC-LIGBT1. Compared with the STA LIGBT, ISM RC-LIGBT has a smaller current peak. It also owns a shorter current tail than that of the SSA LIGBT. This is owing to the better reverse recovery characteristic of ISM RC-LIGBT as illustrated in Fig. 10. During the turn-off period, the ISM RC-LIGBT has the shortest turn-off time, as shown in Fig. 11.

**Fig. 11:** The waveforms of the ISM RC-LIGBT, STA and SSA LIGBT in a complete switching cycle (*L*_C_ = 1mH, *L*_S_ = 1nH, *R*_G_ = 10Ω, *V*_bus_ = 150 V, *N*_A_ = 6 × 10^17^ cm^−3^)

Figure 12 obtains the power loss for the three devices at different frequencies. The total power loss of the RC-LIGBT2 includes the power loss of turn-on/off (*P*_on_/ *P*_off_) and the conduction power loss (*P*_con_). The power loss calculations of the three parts can be given by

3 $$P_{{\text{on/ off}}} = \frac{1}{{t_{{{\text{total}}}} }}\sum\limits_{n = 1}^{N} {E_{{\text{on/ off}}} } { = }\frac{1}{{t_{{{\text{total}}}} }}\sum\limits_{n = 1}^{N} {\int_{t^{\prime}}^{{t^{\prime} + t_{{\text{on/ off}}} }} {V_{{{\text{AK}}}} J_{{\text{A}}} {\text{d}}t} }$$

4 $$P_{{{\text{con}}}} = \frac{1}{{t_{{{\text{total}}}} }}\sum\limits_{n = 1}^{N} {E_{{{\text{con}}}} = \frac{1}{{t_{{{\text{total}}}} }}\sum\limits_{n = 1}^{N} {V_{{{\text{on}}}} J_{{\text{L}}} t_{{{\text{con}}}} } }$$

**Fig. 12:** Power losses under different switching frequencies of the ISM RC-LIGBT, STA and SSA LIGBT at *J*_L_ = 100A/cm^2^ within 1 s

where the summation index *N* corresponds to the times of switching actions in total current commutation time *t*_total_. Here, *t*_on_, *t*_off_ and *t*_con_ represent the time of turn-on/off and the forward conduction. *t*’ is the start time of the three states and *J*_L_ is the loading current density. According to Fig. 12, the ISM RC-LIGBT has the lowest power loss among three types of LIGBTs. Since the *V*_on_ of ISM RC-LIGBT is the smallest among these three devices, as illustrated in Fig. 6, the ISM RC-LIGBT has the lowest *P*_con_. While, with the enhanced injection, the turn-on/off loss of the ISM device does not increase a lot. Therefore, when the operation frequency (*f*_s_) increases to 50 kHz, the power loss of ISM RC-LIGBT still decreases by 29% compared with that of STA LIGBT. Figure 13 compares the power losses with various LIGBTs at the rated *J*_L_ ranging from 100 to 300 A/cm^2^. Although a high density of current leads to an increased power loss, the ISM RC-LIGBT still performs a lowest power loss at *J*_L_ = 300A/cm^2^ among three LIGBTs.

The article "Snapback-Free Reverse-Conducting SOI LIGBT with an Integrated Self-Biased MOSFET" was published in 2022. Journal: Nanoscale Res Lett.

**Fig. 13:** Power losses under different current densities of the ISM RC-LIGBT, STA and SSA LIGBT at *f*_s_ = 50 kHz within 1 s

Figure 14 is key process steps to fabricate the ISM RC-LIGBT. In order to form monocrystalline silicon to fabricate the ISM and NPN**,** the process begins with the silicon direct bonding to form the stack SOI structure. After that, the top SOI region is partly etched, as given in Fig. 14b. Figure 14c–f shows the P-well and N-buffer is formed by implantation and annealing in turn. The N + region of the ISM is implanted together with the N + cathode, which does not require special implantation dose, as denoted in Fig. 14f–h. Finally, the electrodes of cathode, anode and floating ohmic contact are formed by using the same process and mask.

**Fig. 14:** Key process steps to fabricate the ISM LIGBT. **a** Bonding and grinding, **b** part SOI region etching, **c** boron implantation of P-well, **d** phosphorus implantation of N-buffer, **e** anneal, **f** form the gate structure and boron implantation to form P + contact, **g** phosphorus implantation to form N + contact, **h** rapid thermal anneal, **i** formation of electrode

## Conclusion

The ISM RC-LIGBT with an integrated self-biased MOS on the top of the anode active region is proposed and investigated. The novel ISM does not occupy extra device area. By optimizing the parameters of the ISM, the ISM RC-LIGBT could eliminate the snapback effect without degrading the forward conduction characteristic. Meanwhile, the adaptively turned-on ISM provides a current path for reverse-conducting current. The parasitic NPN in the ISM also gives an additional electron extra path during the turn-off and reverse recovery. Thus, the proposed device achieves a better tradeoff relationship between *V*_on_ and *E*_off_, as well as better reverse recovery characteristic. Compared to SSA LIGBT (*L*_b_ = 40/60 μm), it decreases *V*_on_ by 13.3%/20.8% at the same *E*_off_. Moreover, it also features a lower *Q*_rr_ and a better reverse recovery characteristic. Compared to STA LIGBT, the power loss of ISM RC-LIGBT in a completed on/off switching cycle is decreases by 29% at *J*_L_ = 100A/cm^2^, *f*_s_ = 50 kHz. This reveals that the proposed device could reduce the power loss in the application.

The article "Snapback-Free Reverse-Conducting SOI LIGBT with an Integrated Self-Biased MOSFET" was published in 2022. Journal: Nanoscale Res Lett.

## Data Availability

The data used and analyzed during the current study are available from the corresponding authors upon reasonable request.

## Abbreviations

LIGBT: Lateral insulated gate bipolar transistor
SOI: Silicon-on-insulator
SA LIGBT: Shorted anode LIGBT
SSA LIGBT: Separated SA LIGBT
STA LIGBT: Segmented trenches in the anode LIGBT
TBSA LIGBT: Trench barrier shorted anode LIGBT
ISM: Integrated self-biased MOSFET
